# Relationship between Prognosis, Immune Infiltration Level, and Differential Expression of PARVG Gene in Uterine Corpus Endometrial Carcinoma

This article has been retracted.

**DOI:** 10.1155/2022/7376588

**Published:** 2022-05-19

**Authors:** Fei Wang, Juan Bi, Chunxia Yi, Yuan Zhang, Yu Zhang, Qingfang Yue

**Affiliations:** ^1^Department of Gynecology, Shaanxi Provincial People's Hospital, Xi'an 710068, Shaanxi, China; ^2^College of Life Sciences, Northwestern Polytechnic University, Xi'an 710072, Shaanxi, China; ^3^Department of Pharmacy, First Affiliated Hospital, Naval Medical University, Shanghai 200000, China; ^4^University Three Gorges Hospital & Chongqing Three Gorges Central Hospital, Wanzhou, Chongqing, China; ^5^Department of Medical Oncology, Shaanxi Provincial People's Hospital, Xi'an 710068, Shaanxi, China

## Abstract

Endometrial cancer (UCEC) is very common in gynecological diseases and ranks second in the death cause of gynecological cancer in developed countries. The connection between the overall survival of UCEC patients and immune invasion of the tumor microenvironment is positive. The PARVG gene has not been given notice in cancer, and its mechanism is unknown. The research utilized TCGA data to test the function of PARVG in UCEC. The manifestation of PARVG in UCEC was studied by GEPIA. By assessing the survival module, the authors learned the impact of PARVG on the survival of people with UCEC and then obtained UCEC information from TCGA. This study uses logistic regression to prove the possible relationship between PARVG expression and clinical information. From the research of Cox regression, clinicopathological characteristics of people with TCGA were connected with overall survival. Furthermore, the “correlation” module of GEPIA and CIBERSORT was used to study the association between cancer immune invasion and *PARVG*. Using univariate logistic regression analysis with PARVG expression as a categorical variable (median expression value of 2.5), the result suggested that raised PARVG expression was considerably connected with tumor status, pathological stage, and lymph nodes. Multiple factor studies have shown that upregulation of PARVG, distant metastasis, and negative pathological stage are absolute elements of excellent prognosis. In addition, CIBERSORT analysis was utilized to determine that raised PARVG expression has a positive connection with immune infiltration by T cells, mast cells, neutrophils, and B cells. This is recognized in GEPIA's “correlation” module. The above outcomes show us that the raised expression of PARVG is associated with a good prognosis and it raises the proportion of immune cells (such as T cells, mast cells, neutrophils, and B cells) in UCEC. These outcomes tell us that PARVG can be utilized as a possible biomarker to evaluate UCEC's immune infiltration levels and prognosis.

## 1. Introduction

Endometrial carcinoma (UCEC) is a malignant tumor of the endometrial epithelium, known as one of the most frequent gynecological tumors in the world, which poses a serious threat to women's health due to its high mortality rate. Scientists divide endometrial cancer into two types based on biological and histopathological variables [1]. Type II UCECs are nonendometrioid, are more likely to transfer, are always poorly differentiated, and can even be a palindromia after courageous clinical prevention. Conversely, Type I endometrial carcinomas are differentiated well and often endometrioid or carry other risk factors that induce estrogen deficiency, such as obesity [2].

Studies have shown that immune invasion of the microenvironment of the tumor is connected with the lives of lots of people who have cancer. For instance, CD8+ TIL has been confirmed that it is an excellent prognostic element in adenocarcinoma of the lung. It is studied that CD8+ TILs will significantly damage cancer cells in endometrial cancer. In recent years, lots of research on cancer invasion have shown that high presentation of T cells and B cells, like adenocarcinoma B cells, melanoma LCK, breast CD8+ T cells, etc., has an impact on the evaluation of a good integral survival rate for different cancers, such as UCEC. But, as to UCEC, the actual association between prognosis and immune infiltration is unknown.

The PARVG gene at 22q13 has been reported to be deducted in some lines of cancer cells. As a focal adhesion protein, PARVG originates from the parvin group of actin-binding proteins. Because of the deducted presentation of PARVG in some lines of cancer cells and its position at 22q13, it is speculated that PARVG may have a significant influence on the production and growth of oligodendroglioma. In studies of colorectal cancer and breast cancer in recent years, just gene polymorphisms were shown [3]. As a partial and various organ complex, PARVG collects at the position of cell adhesion. PARVG was found to be present in hepatogenic apparatus, and its effect is unknown to people. Leukocyte migration asked that PARVG's ligand integrin-linked kinase possibly be a necessity in the building of cell polarity [4, 5]. For example, PARVG has been confirmed to be associated with renal transplant tolerance [6]. No previous studies have reported a link between PARVG and cancer growth. Nevertheless, the accurate relationship between PARVG and UCEC prognosis was confirmed in our study.

In the public domain, data from The Cancer Genome Atlas (TCGA) is downloaded by us. At the same time, to identify the association of PARVG with prognosis in UCEC, we employed gene expression profiling interactive analysis (GEPIA) and COX regression analysis [7]. The results of this study help us to further understand the possible positive role of PARVG in UCEC, and the underlying correlation and potential works of PARVG-tumor immune interplays are elucidated. Our workflow flow chart is shown in Figure 1. Therefore, PARVG may be a new predictor of prognosis and immune infiltration in patients with UCEC.

## 2. Materials and Methods

### 2.1. Data Acquisition

The authors collected the information of people who have UCEC from the available TCGA in public, which covers 557 cancer tissues. Furthermore, some samples that have inadequate TNM staging information, not including age, integrated survival time, lymph node metastasis, local infiltration, distant metastasis, and TNM staging were subsequently treated. Finally, Cox regression analysis was performed on the remaining 509 cases with clinical data. For identifying PARVG expression's influence on the immune microenvironment, we further analyzed 188 tumor tissues using CIBERSOFT.

### 2.2. Survival and Expression Analysis by GEPIA

In endometrial cancer, the authors evaluated the association in the relation of PARVG presentation and clinicopathological status by looking through the Internet database GEPIA (https://gepia.cancer-pku.cn/index.html) [8]. This website was utilized to study the sequencing presentation of RNA from 522 cancer tissues and 35 healthy cases from GTEx and TCGA. The GEPIA's “survival” model allowed the association of PARVG expression with UCECs prognosis to become available. At the same time, the authors delineated a boxplot with cancer conditions (damaged or healthy) as different to demonstrate the various presentations of PARVG between tissues of cancer and health. The boxplot of clinical with pathological periods as variables was delineated to get to know the PARVG presentation in diverse pathologic periods.

### 2.3. Evaluation of Tumor-Infiltrating Immune Cells

CIBERSORT (https://cibersort.stanford.edu/), a deconvolution algorithm according to gene presentation can assess the variation in the presentation of one group of genes relevant to different genes in the case. TIIC focus can reasonably be accurately evaluated through this period. CIBERSORT's continuous manifestation pushed an increased concentration on cell heterogeneity research [9–11]. The present research tested the ratio of 21 TIICs in UCEC by using CIBERSORT to evaluate its association with survival and molecular subpopulation. Briefly, the standard annotation file formed the gene expression dataset and uploaded it to the CIBERSORT website. There are default signature matrices for 1000 permutation algorithm runs. Through Monte Carlo sampling, the deconvolutional *p* values are estimated by CIBERSORT, and a result confidence measure is formed. 509 TCGA samples were used to evaluate the effect of PARVG expression, which included all genes. Lymphocytes likely to be affected by PARVG were chosen based on a *p* value <0.05. The correlation heat map was used to compare and analyze the relationship between the 21 immune cells. That is the relationship map between each two diverse immune cells in the sample.

Furthermore, the correlation between PARVG expression and possible gene markers was more identified through the “correlation” GEPIA module. Gene markers contained B cells, CD8+ T cells, follicular helper T (Tfh) cells, T-helper 1 (Th1) cells, cells (general), neutrophils, exhausted T cells, natural killer (NK) cells, T-helper 2 (Th2) cells, mast cells, and T-helper 17 (Th17) cells. Earlier research gives clues for the markers of a gene [12–14]. Expression scatterplots of user-defined gene pairs from specific cancer types were plotted with the help of modules relevant to previous studies, as well as the statistical significance of predictions and Spearman's R-values. A relationship map between each of the two various immune cells (correlation heat map) was performed to detect the correlation between the 21 immune cells based on a threshold of *p* value <0.01.

### 2.4. Statistical Analysis

R-3.5.3 analyzed all TCGA statistics. We applied logistic regression, and relationships between clinical features and PARVG expression were analyzed. We performed Cox regression analysis, and the whole survival-related clinical traits were measured. This study treated a *p* value 0.05 as statistically significant. Spearman's R was used to measure the correlation of gene expression, and statistical analysis was also performed. Statistical significance when *p* value <0.01. When the absolute value of R is greater than 0.1, it is considered to correlate.

## 3. Results

### 3.1. Survival Outcomes and Multivariate Analysis

Figure 2 demonstrates a significant association between decreased PARVG expression and worse overall survival (*P* = 0.0015), as shown in Figure 2(a), and advanced pathology (*p* < 0.001), as shown in Figure 2(b). Besides, PARVG was more expressed a lot in tumor specimens than normal (Log2FC < 2, *p* value <0.01), as shown in Figure 2(c).

Table 1 shows Cox regression univariate analysis showed that many factors were greatly related to whole survival, covering pathological stage (HR = 2.32, *p* < 0.001), patient age (HR = 1.02, *P* = 0.42), expression of PARVG (HR = 0.794, *p* value <0.046), and pathological grade (HR = 3.48, *p* value <0.001). Several independent prognostic factors in multivariate analysis, as shown in Table 1 and Figure 3, affecting good prognosis were as follows: younger patient age, upregulated PARVG expression, lower pathological grade, and lower pathological stage. The upregulated PARVG expression, lower patient age, lower pathological stage, and lower pathological grade are independent prognostic factors of favorable prognosis.

### 3.2. Association between PARVG Expression and Clinicopathologic Variables

Deep research is needed on the underlying PARVG expression mechanism. As a result, this study associated it with some clinical areas of UCEC cases and analyzed them. R-3.5.3 analyzed all clinically qualified UCEC cases. In Table 2, it suggested increased PARVG expression was significantly associated with pathological stage using PARVG expression as a categorical dependent variable (median expression value was 2.5) (III vs IV, *p* = 0.039; II vs IV, *p* = 0.038; I vs IV, *p* = 0.012; I-III vs IV, *p* = 0.015).

### 3.3. Relationship between PARVG Expression and Tumor-Infiltrating Immune Cells

Extant findings indicate that tumor-infiltrating lymphocytes have been regarded as individual predictors for the status and survival of the sentinel lymph nodes among patients with cancer [15]. As a result, the researchers endeavor to investigate whether there is a relationship between immune infiltration and PARVG expression in UCEC. Of the total of 509 UCEC samples, the ones with the top one-third and the lowest one-third of expression of PARVG were divided into the group of high expressions and the group of low expressions, respectively. The fraction of 21 types of immune cells in both groups of high and low PARVG expressions was inferred through the exploration of profiles of expressions of the gene from the downloaded samples using an established computational resource, namely CIBERSORT. Eventually, 94 of the samples in the group of high expressions and 94 in the group of low expressions were included due to the inclusion screening criterion.  Figure 4 indicates the results of CIBERSORT.  Figure 4(a) renders the proportions at which the 21 subpopulations of the cells of immunity take up. According to A, macrophages M2, T cells follicular helper, B cells native, Tregs (T cells regulatory), NK cells activated, macrophages M1, T cells CD8, T cells CD8, and macrophages M0 are the primary cells of immunity that were influenced by the expression of PARVG. Of the cells, macrophages M1 (*p* = 0.001), Tregs (T cells regulatory) (*P* = 0.005), T cells CD8 (*P* = 0.002), NK cells activated (*P* = 0.252), NK cells activated (*P* = 0.008), macrophages M2 (*P* = 0.217), T cells follicular helper (*P* = 0.005), and T cells CD8 (*P* = 0.049), all account for a larger proportion in the group of high expression than that in the group of low expression. On the contrary, the proportion of T cells CD8 (*P* = 0.002), B cells native (*P* = 0.135), and macrophages M0 (*P* = 0.251) appears to be explicitly lower. Moreover, as Figure 4(b) revealed, the heatmap of correlation showed the correlation of the proportions among different t TIIC subpopulations was weak to moderate.

The module of “correlation” of GEPIA unveiled the connection between the expression of PARVG and markers of the gene among various types of tumor-infiltrating cells of immunity, such as B cells, mast cells, neutrophils, and DCs, as well as various functional T cells, including Tfh, Th1, Tregs, Th17, Th2, and exhausted T cells, as shown in Table 3. According to the results, the expression of PARVG has relationships with over 50% of the marker sets among various cells of immunity in UCEC. The markers of genes that were influenced by the expression of PARVG were STAT4 of Th1, IL13 of Th2, KIR2DL4, STAT3, GATA3, IL17A of Th17, KIR2DL1, CD79A of B cells, STAT5A, KIR2DS4 of natural killer cells, CTLA4, KIR2DL2, CCR7 of neutrophils, STAT6, BCL6 of Tfh, and LAG3 of T cell exhaustion, as well as TPSB1 and TPSB2 of mast cells. Spearman's correlation coefficients were adopted to calculate the correlations. The results between PARVG and neutrophils, NK cells, markers of B cells, T cells, and mast cells shared similarities with CIBERSORT. As a result, the findings indicate PARVG plays a possibly critical role in the regulation of the richness of NK cells, mast cells, neutrophils, B cells, and T cells.

## 4. Discussion

PARVG was only reported in previous studies [6] to exist in transplanted kidney tolerance. Here, we found that changes in levels of expressions of PARVG had correlations with a prognosis of UCEC. The results suggest that upregulation of PARVG is an independent variable of prognosis for a positive prognosis. Also, according to the result of multivariate analysis, a surge in PARVG expression was significantly correlated with the patient's age, pathological stage, pathological grade, and other clinical characteristics. In addition, different groups of the markers of immunity and criteria of infiltration of immunity had correlations with the expression of PARVG in UCEC. As a result, as shown in previous research, PARVG could have an impact on the immunity of tumors and potentially be adopted as a capable biomarker for cancer.

The present study found a relationship between the expression of PARVG and levels of infiltration of immunity in UCEC. According to the analysis of CIBERSORT, there was a substantial explicit correlation between the expression of PARVG and the infiltration levels of mast cells, neutrophils, NK cells, B cells, and T cells in UCEC. Similarly, the connection between markers of genes of various cells of immunity and the expression of PARVG concerned the importance of PARVG in the regulation of the microenvironment of immunity of tumors in UCEC. To begin with, the proportions of NK cells, several types of T cells, mast cells resting, and B cells, had obvious increases in the group of high expressions than those in the group of low expressions based on an algorithm of CIBERSORT. Besides, the module of “correlation” of GEPIA has been applied to confirm the discovery. CD79A of B cells showed a positive relationship with the expression of PARVG. The finding indicated that PARVG could regulate plenty of B cells in tumors. Tfh, Th1, Th17, and Th2 are various T cells with functions. The surge in the expression of PARVG has positive relationships with their markers, including CTLA4, GATA3, IL13, STAT4, STAT3, STAT5A, IL17A, STAT6, BCL6, and LAG3. The relationships were indicators of a potential device at which PARVG plays a regulatory role in the functions of T cells in UCEC. Additionally, significant relationships were found between neutrophil markers and PARVG and mast cells. According to previous reports, M1 macrophages and Tregs have the most occurrence and account for the largest proportion of the composition of cells of immunity in endometrial carcinoma [16]. T cells with high expressions and signatures of B cells have relationships with the entire extended survival assumed in different kinds of tumors, such as breast cancer [15]. Combined with the results, PARVG is critical to recruiting and regulating cells of infiltration of immunity in UCEC.

According to the analysis of CIBERSORT, the expression of PARVG had a significant relationship with the levels of infiltration of neutrophils, T cells, B cells, mast cells, and NK cells in UCEC. However, the connection between the markers of genes of various cells of immunity and the expression of PARVG shows PARVG is critical to the regulation of the microenvironment of immunity of UCEC tumors. To start, the proportion of several T cells, NK cells, B cells, and mast cells resting had a significant surge in the group of high expressions than those in the group of low expressions according to the result of the CIBERSORT algorithm. Besides that, the module on “correlation” of GEPIA supported the result. B cell CD79A was positively correlated with PARVG expression. It can be said that PARVG potentially plays a role in regulation in numerous B cells regarding tumors. The Th2, Th17, and Th1, are T cells that have various functions. The improved PARVG expression has positive relationships with their markers GATA3, IL13, STAT4, IL17A, STAT3, STAT5A, STAT6, BCL6, CTLA4, and LAG3. The relationships can be a device by which the regulation of PARVG applies to T cell function in UCEC. In addition, markers of neutrophils and mast cells were significantly associated with PARVG. According to previous reports, Treg and M1 macrophages are the most common in endometrial carcinoma [16] and dominate the composition of immune cells. High expression of signatures of T and B cells has correlations with overall survival that has been extended, which has been assumed among several tumors such as breast cancer [15]. It can be seen that PARVG is the key to recruiting and regulating cells of infiltration of immunity in UCEC.

Some of the research on the TIIC's function in human tumors have generally concentrated on T cells, reporting their responses to immune checkpoint inhibition and their survival [17–20]. Complementing the combined literature, T cells were identified as a positive prognostic aspect in this study. An important breast cancer evolvement regulator was shown to be tumor-infiltrating B cells, according to another study [21]. Between histological subtypes and stages, breast cancer development concentrations of varied tumor-infiltrating B lymphocytes (TIBs) can be seen in the overall process of breast cancer development. A significant function in breast cancer evolvement has been indicated in B cells [22]. B cells insinuate, grow, and evolve in tumors motivated by signals in the microenvironment. By secreting tumor-specific antibodies by TIB, T cell responses were improved, and the structure and function of TLS were sustained. Anti-tumor immune functions were exerted, and all related to helpful results in breast cancer [21,23,24]. As a result, the good impact of PARVG on UCEC is similar to the impact of higher T cells and B cells abundance, suggesting a working principle by which PARVG may affect UCEC's whole survival.

There are currently no studies that correlate PARVG expression with T cell good prognosis and immune infiltration. The appearance and growth of tumors may have the participation and role of parvin's, and studies have presented that its function is associated with tumor inhibition genes [25,26]. A decrease in PARVG expression was presented in some cancer cell lines, according to a supporting hypothesis by Korenbaum et al. [27]. Nevertheless, it is worth saying that the promoter sequence remains unclear and the mechanism leading to the inactivation of abnormally hypermethylated genes at the PARVG gene promoter has not been assessed [28].

In conclusion, there is a correlation between enhanced PARVG expression and a good prognosis. At the same time, different proportions of UCEC immune cells affect the expression of PARVG, such as NK cells, B cells, T cells, neutrophils, and mast cells. Therefore, PARVG plays an important role in immune infiltration and may be used as a prognostic biomarker of UCEC.

## Figures and Tables

**Figure 1:** Workflow of our study.

**Figure 2:** Survival outcome and expression difference analyzed by GEPIA. (a) Increased PARVG expression is associated with a favorable outcome. (b) Differential expression of PARVG in different disease states (tumor or normal). (c) Differential expression of PARVG in the different pathological stages.

**Figure 3:** Multivariate Cox analysis of PARVG expression and other clinicopathological factors.

**Figure 4:** PARVG-related immune infiltration alteration. (a) T cells CD8 (*P* = 0.049), NK cells activated (*P* = 0.008), T cells CD8 (*P* = 0.002), T cells follicular helper (*P* = 0.005), T cells regulatory (Tregs) (*P* = 0.005), NK cells activated (*P* = 0.252), macrophages M1 (*P* = 0.001), and macrophages M2 (*P* = 0.217) share a higher proportion in high expression group compared with low expression group. In contrast, the proportions of B cells native (*P* = 0.135), T cells CD8 (*P* = 0.002), and macrophages M0 (*P* = 0.251) are apparently lower. (b) The proportions of different TIICs subpopulations were weakly to moderately correlated.

**Table 1:** The results of Cox regression analysis.

Clinicopathologic variable	HR (95% CI)	*p*
AGE ≤64		
Age	1.02 (0.97–1.08)	0.42
Stage	2.32 (1.49–3.19)	<0.00
Grade	3.48 (1.74–6.95)	<0.00
PARVG	0.44 (0.20–0.95)	0.04
AGE >64		
Age	1.04 (1.00–1.09)	0.07
Stage	1.81 (1.41–2.33)	<0.00
Grade	1.86 (1.12–3.11)	0.02
PARVG	0.56 (0.31–1.01)	0.05

Univariate analysis using Cox regression revealed that some factors, including patient age (HR = 1.02, *p* value = 0.42), pathological stage (HR = 2.32, *p* value <0.001), and pathological grade (HR = 3.48, *p* value <0.001) along with the expression of PARVG (HR = 0.794, *p* value <0.046) are significantly associated with overall survival. The upregulated PARVG expression, lower patient age, lower pathological stage, and lower pathological grade are independent prognostic factors of favorable prognosis.

**Table 2:** Association between PARVG expression and clinicopathologic variables using logistic regression.

Clinical characteristic	Total (N)	The odds ratio in PARVG expression	*p*
Age (continuous)	509	0.888 (0.628–1.258)	0.505
Stage (III vs IV)	139	0.351 (0.130–0.949)	0.039
Stage (I vs IV)	343	0.296 (0.114–0.765)	0.012
Stage (II vs IV)	75	0.321 (0.109–0.939)	0.038
Stage (I–III vs IV)	509	0.311 (0.121–0.796)	0.015

**Table 3:** Correlation analysis between PARVG expression and gene markers of B cells, natural killer (NK) cells, neutrophils, T-helper 1 (Th1) cells, T-helper 2 (Th2) cells, follicular helper T (Tfh) cells, T-helper 17 (Th17) cells, exhausted T cells and mast cells via “correlation” module of GEPIA.

Description	Gene markers	UCEC			
		Tumor		Normal	
		R	*p*	R	*p*
B cell	CD79A	0.254^∗∗^	<0.000	0.435^∗∗^	0.009

Natural killer cell	KIR2DL1	0.08	0.059	0.491^∗∗^	0.003
	KIR2DL3	0.075	0.078	0.390^∗^	0.021
	KIR2DL4	0.292^∗∗^	<0.000	0.754^∗∗^	<0.000
	KIR3DL1	0.102^∗^	0.016	0.534^∗∗^	0.001
	KIR3DL2	0.099^∗^	0.02	0.515^∗∗^	0.002

^∗^ *P* < 0.05, ^∗∗^*P* < 0.01, ^∗∗∗^*P* < 0.001.

## Data Availability

The simulation experiment data used to support the findings of this study are available from the corresponding author upon request.
